The article "Intelligent Reconstruction Algorithm-Based Computed Tomography Images for Automatic Detection of Gastric Tumor" was published in 2022. Journal: Comput Math Methods Med.

# Intelligent Reconstruction Algorithm-Based Computed Tomography Images for Automatic Detection of Gastric Tumor

**DOI:** 10.1155/2022/8179766

**Published:** 2022-06-28

**Authors:** Yuanyuan Zhang, Lisha Chen, Huixin Chen

**Affiliations:** Department of Digestive Diseases, Huizhou Municipal Center Hospital, Huizhou, 516001 Guangdong, China

## Abstract

The aim of this study was to explore the application of computed tomography (CT) images in the diagnosis of gastric tumor under the intelligent reconstruction algorithm (IRA). 120 patients with gastric cancer were selected and all the patients underwent CT scanning, and CT images were analyzed based on the Feldkamp-Davis-Kress algorithm (FDK algorithm) to evaluate the imaging features of gastric lesions. According to biopsy or surgical pathology, the detection rate of CT images was calculated. The results showed that there were three pathological types of benign tumors (polyps, leiomyomas, and mesenchymomas) and three pathological types of malignant tumors (mesenchymomas, adenomas, and lymphomas). In addition, the detection rates of CT scans were different, reaching 94.2% on different orientations of the stomach, 90.7% of benign tumors, and 90.9% of malignant tumors, so the detection rate of different orientations was relatively high. CT images based on the FDK IRA could realize a high detection rate in diagnosis, accurately locate the lesion, and display the characteristics of the lesion and the metastasis of surrounding tissues; there were significant differences between benign and malignant gastric tumors in CT images, and the detection effect was obvious, which is worthy of clinical application and promotion.

## 1. Introduction

Stomach tumor is one of the common tumors in the digestive tract. Most gastric tumors are mainly malignant tumors, such as lymphomas and mesenchymomas [1], and a small number are benign tumors, such as gastric adenomas and gastric polyps. The benign tumors can be cured by endoscopic submucosal biopsy or submucosal resection, and it is recommended that patients undergo resection to achieve radical cure even if benign tumors grow to a certain stage. However, for malignant tumors, it has to judge whether there is abdominal metastasis based on the results of imaging examinations, and finally determine the treatment method [2]. Using X-rays, gamma (*γ*) rays, and ultrasound, CT can scan a certain part of the human body together with a highly sensitive detector. It is featured with fast scanning time and clear scanned images [3]. The imaging principle is to use energy rays to scan the object, rely on projection data obtained from the outside of the object, and present tomographic imaging of the inside of the object in the form of two-dimensional (2D) or three-dimensional (3D) images with a specific reconstruction algorithm [4].

In recent years, CT imaging has been widely used in the field of medical clinical diagnosis for tomography on the injured parts of the human body. The disease can be determined by analyzing the images. CT examination has become an indispensable way in the medical field to diagnose the stomach [5]. With the continuous update of the 3D cone beam reconstruction algorithm, the FDK algorithm proposed by Feldkamp [6] is relatively prominent. Although this algorithm can only obtain good reconstruction results when the reconstruction cone angle is small, it has the advantages of simple operation, effective method, and convenience operation in practical application projects, so the FDK algorithm has always been the main algorithm used in practical projects. In this study, CT images based on the FDK algorithm were adopted to examine the stomach, which can effectively find the smaller lesions, increase the detection rate of gastric tumors, and help early detection and timely diagnosis and treatment of gastric tumors [7–9].

In summary, the CT images based on FDK algorithm were adopted to evaluate different parts of the stomach and different types of gastric tumors to observe the different pathological characteristics of gastric tumors, so as to provide a reference for its clinical diagnosis.

## 2. Materials and Methods

### 2.1. Selection of Research Objects

120 patients with different types of gastric tumors in the hospital from May 10, 2018, to May 10, 2020, were selected in this study, including 86 males and 34 females, with an average age of 45.7 ± 6.9 years old. This study had been approved by the ethics committee of the hospital. Besides, all patients and their families had understood the situation of the study and signed the informed consents.

Inclusion criteria: patients with gastric tumors diagnosed by clinical and CT examination; patients older than 75 years old; patients without contraindications to CT scanning; and patients without resection of gastric tumor before.

Exclusion criteria: patients with mental illness; patients with other malignant tumors; patients with incomplete basic clinical data; and patients with poor quality of CT image.

### 2.2. Observation Parts and Indicators

The characteristics of the lesions of 120 patients were analyzed comprehensively. The sites that underwent with CT imaging examination included gastric antrum, cardia, gastric fundus, and gastric body according to the structure of the stomach; or forearm, greater curvature side, posterior wall, and minor curvature side according to the orientation; or the round, quasi-circular, diffuse thickened, and irregular according to the shape; or cystic degeneration, calcification, and necrosis according to the internal characteristics. In addition, it should determine the maximum diameter of the lesion based on the size, if there was any surrounding tissue invasion or metastasis, and if it could be reinforced with scanning enhancement technology. It should be judged based on biopsy or surgical pathology, and the CT image detection rate under IRA was calculated based on the diagnosis results.

### 2.3. CT Examinations of Patients

CT scanner was used for CT examination. A total of 120 patients underwent the enhanced scans for 3 phases. Before the CT examination, the patient was required to fast for 4 to 6 hours and take 500 mL of warm water orally half an hour before the examination. The patient was injected with 15 mg of 654-2 intramuscularly 10 minutes before the scan, and then took 50 mL of warm water orally 3 minutes before the examination to ensure hypotonic filling of the gastric cavity. The patient was scanned from the top of the diaphragm to the level of the pelvic entrance. The scanning parameters were defined as follows: the tube voltage was 120 kV, the tube current was 100-250mAs, the image thickness was 5.00-7.00 mm, the scanning interval was 0.5 mm, the pitch was 0.984 : 1, and the matrix was 512 × 512. The enhanced scanning was realized by injecting 300 mg/mL contrast agent (Electropromide Injection) at 3 mL/s with the injection dosage of 1.5 mL/kg. After the injection of the contrast agent, the patient was scanned in the arterial phase, portal vein phase, and delayed phase at 30s, 50s, and 120 s, respectively.

### 2.4. Calculating Steps of FDK Algorithm

The FDK algorithm mainly included three steps: weighting of projection data, one-dimensional (1D) filtering, and back projection.

**Step 1 .**

The projection data of each division was weighted using a function similar to the cosine function, and the distance and angle difference of the voxel source point were appropriately corrected. The calculation equation was given as follows:

(1) $$\begin{array}{c} {\text{D}}_{\Phi }^{\prime }\left(\omega ,\Phi \right)=\frac{h}{\sqrt{h^{2}+A^{2}+B^{2}}}D_{\Phi }\left(A,B\right). \end{array}$$

In the above equation (1), *A* and *B* represented voxels. *D*_*Φ*_(*A*, *B*) represented the projection data, and D_*Φ*_′(*ω*, *Φ*) represented the weighted projection data.

**Step 2 .**

The weighted projection data was transformed in the horizontal direction firstly (as equation (2) below), and then the projection data with different projection angles was filtered with the horizontal 1D frequency domain (as shown in equation (3) below):

(2) $$\begin{array}{c} {\text{D}}_{\Phi }^{*}\left(\omega ,\Phi \right)=\int_{-\infty }^{+\infty }D_{\Phi }\left(A,B\right)e^{-i\omega B}d\omega , \end{array}$$

(3) $$\begin{array}{c} {\overset{\sim }{D}}_{\Phi }\left(A,B\right)=\int_{0}^{\infty }\omega D_{\Phi }^{*}\left(\omega ,\Phi \right)e^{i\omega B}d\omega . \end{array}$$

In the above equations, D_*Φ*_^∗^(*ω*, *Φ*) represented the projection data after Fourier transform, *ω* represented the filter function, and ${\overset{\sim }{D}}_{\Phi }\left(A,B\right)$ referred to the projection data after frequency filtering.

**Step 3 .**

The 3D back projection was performed along the X-ray direction. The reconstructed voxel was the sum of projection angles of all rays passing through the pixel, and the equations were defined as follows:

(4) $$\begin{array}{c} A\left(m\right)=m\cdot \overset{\wedge }{a}\frac{h}{h+m\cdot \overset{\wedge }{x^{\prime }}}, \end{array}$$

(5) $$\begin{array}{c} B\left(m\right)=m\cdot \overset{\wedge }{b}\frac{h}{h+m\cdot \overset{\wedge }{x^{\prime }}}, \end{array}$$

(6) $$\begin{array}{c} g\left(m\right)=\frac{1}{4\pi^{2}}\int \frac{h^{2}}{{\left(h+m\cdot \overset{\wedge }{x^{\prime }}\right)}^{2}}{\overset{\sim }{D}}_{\Phi }\left[A\left(m\right),B\left(m\right)\right]d\Phi . \end{array}$$

Equations (4) and (5) were the coordinates of the point of the voxel in the coordinate system mapped to the virtual area detector coordinate system. Equation (6) referred to the back projection. *A*(*m*) and *B*(*m*) represented the coordinates of the voxel in the coordinate system of virtual area detector, and they were calculated by the computer through interpolation. Since the back projection design was independent in each division, the *g*(*m*) could be calculated with accumulation in the computer.

### 2.5. Simulation Experiment

The reconstruction effects of FDK, SS-FDK (short scan FDK), and our algorithm are compared through experiments [10].  Table 1 shows simulation parameters.

### 2.6. Statistical Methods

The data processing in this study was analyzed by SPSS19.0 version statistical software, the measurement data is expressed by mean standard deviation ($\bar{x}\pm s$), and the counting data is expressed by percentage (%). The basic data of the patients were counted, and the detection rate was calculated. The difference was statistically meaningful at *P* < 0.05.

## 3. Results

### 3.1. Simulation Results

In the simulation, the number of detector sampling points *N* is set to 256, and the size of the reconstructed image is set to 256 × 256 in the test. The number of detector channels *N* =256, the number of sampling points 256, the distance from the source to the center of rotation 44, the distance from the source to the center of the detector 88, and the length of the virtual detector 2 are set. The results of CT image processing by FDK, SS-FDK, and this algorithm is shown in Figure 1.

### 3.2. Statistical Results for Basic Information

Among the 120 patients, 58 cases (48.3%) suffered from abdominal pain and bloating, 29 cases (24.2%) had decreased appetite and malaise, 21 cases (17.5%) suffered from nausea and vomiting, 12 cases (10.0%) had upper gastrointestinal bleeding, and 6 cases (5.0%) were found during physical examination. The basic calculation data of the patients is shown in Figure 2. In terms of gastric tumor classification, there were 54 patients with benign tumors and 66 patients with malignant tumors. The specific ratio is shown in Figure 3.

### 3.3. CT Imaging Characteristics of Benign Tumors

Leiomyoma in benign tumors was one of the gastrointestinal mesenchymal tumors (GIMTS) in the esophagus, and it was rate in the stomach. The main CT manifestations were uniform low-density lesions, commonly growing in the cavity. After enhancement, they showed mild or moderate enhancement, and mucosal line was complete (Figure 4(a)). Mesenchymoma was the most common mesenchymal tumor of the gastrointestinal tract, which could be found in any part of the gastrointestinal tract. Mesenchymomas were potentially malignant. The typical CT image showed that the growth pattern of the lesion could be extraluminal, intraluminal, and mixed. When the mass was large, internal hemorrhage and necrosis were common, and the growth showed uneven enhancement, showing high, isodense, or low density, respectively; in addition, the mucosal line on the surface of the lesion was complete, and occasional calcification inside the tumor could be found sometimes (Figure 4(b)).

### 3.4. CT Imaging Characteristics of Malignant Tumors

Gastrointestinal tract was the common site of extranodal lymphomas. CT images showed thickened stomach body, fundus, and gastric wall. It mainly included the diffuse thickening, segmental, and limited thickening. The density of lesions was generally uniform. Necrosis was rare, and even mild enhancement could be seen after enhancement. The gastric wall was expanded to a certain degree, and the gastric wall mucosal line was continuous or interrupted, as indicated by the arrow in Figure 5.

Heterotopic pancreas, also known as vagus pancreas, was a solitary pancreatic tissue that grew outside the anatomical part of the normal pancreas. There was no anatomical or vascular connection with the normal pancreas. Ectopic pancreas occurred mostly in the gastrointestinal tract, and about 70%-86.5% were in the stomach, duodenum, and proximal jejunum. The prevalence age was 40-60 years old. It was more common in men. Most patients had no obvious symptoms and were usually found accidentally by surgery or biopsy. Its typical CT findings included soft tissue masses located in the submucosa, uniform density on plain scan, rare hemorrhage, necrosis, and calcification, and even cystic change. The lesions were oval, lobulated, or irregular, and the length and diameter were mostly less than 4 cm. Most of the lesions were found out of the cavity. The enhancement degree of the enhanced scan focused varies greatly depending on the composition of the heterotopic pancreas. The pancreatic acinar tissue was the main focus, and the enhancement was obvious; while the pancreatic duct and proliferating smooth muscle were the main focus, the enhancement was not obvious. The central umbilical fovea sign was characteristic for the diagnosis of heterotopic pancreas.

### 3.5. CT Image Analysis of Different Gastric Lesions

Images of 120 patients with gastric tumors were analyzed by two associate chief physicians with more than 20 years of work experience using the double-blind method. The tumor shape, size, margin, tumor density, growth mode, enhancement, and metastasis were observed. 7 cases were not found due to small or concealed affected side. The number of cases found on the side of the small bend was large. The specific data of the lesions are illustrated in Figure 6.

### 3.6. Analysis of Gastric Benign Tumor Based on CT Image

Gastric benign tumors were mainly divided into two categories, adenomas or polypoid adenomas originating from the epithelial tissue of the gastric mucosa, and the leiomyomas, fibroids, neurofibromas, lipomas, and hemangiomas derived from the mesenchymal tissue of the stomach wall. Symptoms of gastric benign tumors were rarely seen. Some complications or malignant changes could be found due to large tumors. Common complications included benign tumors near the cardia, which may eventually cause dysphagia. Most of them resolved spontaneously, and a few may have congestion, edema, even intussusception, necrosis, perforation, and peritonitis. In addition, ulcers, gastric discomfort, pain, and even bleeding, leiomyomas, and neurofibromas could cause acute hemorrhage. In this study, 54 cases of benign tumors mainly included polyps, leiomyomas, and mesenchymomas, all of which showed clear contours, no gastric wall, no surrounding tissue invasion, and no surrounding lymph nodes. The specific classification of benign tumors is disclosed in Figure 7.

### 3.7. Analysis of Gastric Malignant Tumor Based on CT Image

Gastric malignant tumors were particularly prone to metastasis and recurrence. It could be divided into gastric cancer, malignant lymphomas, and malignant mesenchymomas according to their different origins. Gastric cancer originated from epithelial cells of gastric mucosa, gastric malignant lymphomas originated from lymphoid tissue, and gastric malignant mesenchymomas originated from mesenchymal tissue. Among them, the gastric cancer was the most common, accounting for the largest proportion of malignant tumors of the digestive tract. When the tumor grew to a certain extent, there would be pain and discomfort in the gastric cavity, nausea, poor appetite, bleeding, anemia, weight loss, and even cachexia. The treatment effect was poor. In this study, 66 cases of malignant tumors included malignant mesenchymomas, adenomas, and lymphomas. The main manifestations were blurred contours, no stomach wall, invasion of the stomach wall by surrounding tissues, and organs or lymph nodes for metastasis. The specific detection status is shown in Figure 8.

### 3.8. Detection Rate of CT Image in Different Sites and Malignant and Benign Tumors

CT images based on IRA had different detection rates for different sites of gastric tumors, benign tumors, and malignant tumors. The specific detection conditions are disclosed in Figure 9.

### 3.9. Detection of Multiple Sites of Benign Tumors

Benign tumors were detected in different structural parts of the stomach. The data showed that polyps were found to be more common in the gastric body and antrum. They were round or oval soft tissues with uniform density and smooth surface (Figure 10); leiomyomas were more common in the stomach body, and it was mostly circular or quasi-circular, with clear borders. What's more, the enhanced scan was slightly or moderately enhanced (Figure 11).

### 3.10. Detection of Multiple Sites of Malignant Tumors

Mesenchymoma was a rare clinical tumor, which could be found at both ends of the muscular layer of the stomach wall. It grew along the vertical direction of the stomach wall. The tumor was large but relatively suffered from limited growth. The tumor was mostly the round or quasi-circular soft tissue masses that grow outside, inside, and both inside and outside the cavity, with ulcer formation on the surface. Tumor had abundant blood supply, and progressive enhancement was the main enhancement method of gastric mesenchymomas. The diameter of malignant mesenchymomas was more than 5 cm, the shape was not regular, the mass density was more uneven, and it was accompanied by hemorrhage, necrosis, cystic change, with unclear boundary with the surrounding organs or tissues. In this study, mesenchymomas were more common in the fundus and body of the stomach, and they grew vertically along the gastric wall. The gastric wall had normal softness and uniform density. The enhanced scan showed uniform enhancement. The multiple sites of mesenchymomas are shown in Figure 12.

Gastrointestinal lymphomas originated from lymphomas of the gastrointestinal tract, including gastric lymphomas, small intestinal lymphomas, immunodeficiency-related lymphomas, and other lymphomas, which were relatively rare. In this study, gastrointestinal lymphomas were more common in the gastric antrum and gastric body with non-Hodgkin lymphomas. It was mostly manifested as diffuse thickening of the stomach wall, but with a certain degree of flexibility and expansion; the density was not uniform, with mild or moderate enhancement; 2 cases were found with invaded the tissues around the stomach, 5 cases were accompanied with invaded the external gastric lymph nodes, and 9 cases were with invaded the entire stomach in multiple locations.

Gastric cancer mostly originated from mucosal epithelial cells on the surface of the gastric wall, mainly reflected as the gastric adenocarcinoma. Gastric adenocarcinoma arose from malignant transformation of gastric gland cells. It was a malignant tumor with the highest incidence in the gastrointestinal tract. In this study, gastric adenocarcinoma mostly occurred in the antrum of the stomach. The gastric wall showed varying degrees of irregular thickening and stiffness. Invasive extension could be found along the stomach wall, the shape of the gastric cavity was fixed but narrow, and the enhanced scan showed moderate and obvious enhancement. 6 cases showed soft tissue masses with uneven density, and the degree of enhancement was lower than that of invasive gastric cancer. 12 cases had enlarged lymph nodes, and 4 cases had multiple site invasion.

## 4. Discussion

Due to the various types of stomach cavities, the gastric mucosa was flexible and frequently peristaltic. CT scan images routinely used in medicine were prone to false thickening of the stomach wall and obvious motion artifacts, so it was difficult to find small lesions and occult lesions. Among the various 3D cone beam CT approximate reconstruction algorithms, the FDK algorithm is the main method currently applied in practice [11]. The FDK algorithm was adopted in this study, which could effectively expand the gastric cavity, made it smooth and relax, and helped eliminate artifacts caused by gastric wall peristalsis. It indicated that the CT image scan results based on the FDK algorithm were indeed better than those of the conventional scan methods.

Leiomyoma is one of GIMTS of the esophagus. Most of them are uniform low-density lesions, which are slightly enhanced after enhancement. The mucosal line on the surface of the lesion is intact. Slattery JM et al. found that gastroscopy could not detect leiomyomas [12]. CT examination in this study could clearly show the shape of the tumor and evaluate the expansion of the tumor into or out of the cavity. Thus, the inspection method of this study was superior. Gastrointestinal mesenchymomas can be found in any part of the gastrointestinal tract. The growth of the lesion can be seen in the cavity, out of the cavity, or mixed type. After enhancement, it shows uneven enhancement. The mucosal line on the surface of the lesion is complete. Sun et al. [13] believed that mesenchymomas were potentially malignant, and had the following characteristics: the tumor grew out of the cavity; the maximum diameter of the tumor was more than 5 cm; the tumor had cystic transformation or necrosis; the tumor was calcified; and it invaded surrounding tissues or metastasizes to distant organs, this is similar to this article. In recent years, many scholars have pointed out [14–16] that CT imaging based on IRA did have a good advantage in showing the location of the lesion, the shape of the mass, and the spread and metastasis. Gastrointestinal lymphoma is one of the common extranodal lymphomas, which is mainly manifested as diffuse thickening of the fundus, body, and wall of the stomach, with uniform lesion density, and even mild enhancement after enhancement. The results of this study were consistent with the results reported by Thieblemont et al. [17]. At present, there are many medical diagnosis methods for gastrointestinal lymphomas. The CT impact assessment using IRA is the most applied and the most comprehensive method [18].

With the rapid update of electronic information technology in recent years, CT examination has become more and more widely used in the diagnosis of gastrointestinal diseases and has now become one of the most accurate examination methods for location and staging of gastric tumor [19–21]. CT scan based on the FDK algorithm has become an effective supplement to routine examinations, which can effectively locate the gastric tumors and preoperative staging, thereby having reliable clinical reference significance.

## 5. Conclusion

CT imaging based on FDK algorithm was adopted to scan and evaluate the different structures, different orientations, and different types of tumors in the stomach. CT images based on the FDK IRA could realize a high detection rate in diagnosis, accurately locate the lesion, and display the characteristics of the lesion and the metastasis of surrounding tissues; there were significant differences between benign and malignant gastric tumors in CT images, and the detection effect was obvious, which is worthy of clinical application and promotion. The limitations of this study lied in that the small, flat, or hidden lesions were limited to be observed, and the color of the lesion could not be accurately distinguished. All in all, CT images based on image enhancement algorithms in this study effectively compensated for the conventional CT examinations, and had obvious advantages in the location and staging of gastric tumor, and reduced the FNR and FPR for clinical diagnosis of gastric tumors.

## Figures and Tables

**Figure 1:** Comparison of reconstruction effects of three algorithms. (a) FDK algorithm; (b) SS-FDK algorithm; (c) this research algorithm.

**Figure 2:** Statistical results for basic information of patients. A, B, C, and D referred to abdominal pain, decreased appetite, nausea, and upper gastrointestinal bleeding, respectively, while E indicated the number of patients whose tumor was found occasionally.

**Figure 3:** The specific ratio of benign tumor and malignant tumor.

**Figure 4:** CT images of leiomyoma and mesenchymal tumor. (a) CT image of leiomyomas (low-density lesion with complete mucosal line); (b) CT image of mesenchymomas (internal bleeding with uneven enhancement).

**Figure 5:** CT image of lymphomas. The white arrow suggested the lesion with even density and continuous mucosal line.

**Figure 6:** The specific sites of CT examination. A: forearm; B: rear arm; C: large bend side; D: small bend side; and E: multiple parts. ∗Compared with the small bend side, *P* < 0.05.

**Figure 7:** Detected types of benign tumors.

**Figure 8:** Detected types of malignant tumors.

**Figure 9:** Detection rate of CT image on different gastric tumors.

**Figure 10:** Number of detected polyps in various sites. ∗Compared with the gastric body, *P* < 0.05.

**Figure 11:** Number of detected leiomyomas in various sites. ∗Compared with the gastric body, *P* < 0.05.

**Figure 12:** Number of detected mesenchymomas in various sites. ∗Compared with the gastric body, *P* < 0.05.

**Table 1:** Simulation parameters.

Project	Parameter
Scanning radius	260 mm
Distance from source to detector	400 mm
Projection angle sampling interval	1°
Maximum cone angle	±8°
Maximum fan angle	±28.5°
Array rows	45
Number of detector columns	175
Detector unit size	2.5 mm ×2.5 mm
Reconstructed image size	256 × 256
Pixel size	1 mm ×1 mm

## Data Availability

The data used to support the findings of this study are available from the corresponding author upon request.
